# A Bibliometric Analysis of Scientific Research Publications Related to Pesticide Poisoning in the South Asian Countries

**DOI:** 10.7759/cureus.38134

**Published:** 2023-04-25

**Authors:** Prateek Pandey, Swarupa Chakole, Mayur B Wanjari, Roshan Prasad

**Affiliations:** 1 Department of Medicine, Jawaharlal Nehru Medical College, Datta Meghe Institute of Higher Education and Research, Wardha, IND; 2 Department of Community Medicine, Jawaharlal Nehru Medical College, Datta Meghe Institute of Higher Education and Research, Wardha, IND; 3 Department of Research and Development, Jawaharlal Nehru Medical College, Datta Meghe Institute of Higher Education and Research, Wardha, IND; 4 Department of Medicine and Surgery, Jawaharlal Nehru Medical College, Datta Meghe Institute of Higher Education and Research, Wardha, IND

**Keywords:** pesticide control, south asian countries, bibliometric analysis, regulations, suicide, pesticide self-intoxication

## Abstract

Pesticide self-intoxication leading to suicide is a widespread phenomenon in India. Implementing regulations prohibiting the use of highly toxic pesticides in agriculture has proven effective in reducing the overall suicide rate in various South Asian countries without compromising agricultural production. In this study, we conducted a bibliometric analysis of scientific publications on pesticide poisoning in South Asian countries using various databases, including PubMed, Scopus, and Web of Science, using relevant Medical Subject Heading (MeSH) terms. To analyze the data, we employed R Studio and Microsoft Excel 2019, which enabled us to collect information on the number of scientific publications, citation frequency, and keyword trends. Our analysis involved 417 articles, and the results indicated a crucial need for greater awareness and improved management of pesticide poisoning in South Asian countries. Our findings provide valuable insights for policymakers and offer guidelines for pesticide control.

## Introduction and background

Over the last few decades, agricultural pesticides have become increasingly prevalent in rural areas of developing countries. The accessibility of these pesticides has, unfortunately, made them a common choice for individuals who attempt to inflict self-harm through poisoning [1]. The global impact of pesticide poisoning is significant and has become a leading cause of illness and death [2]. It is estimated that approximately three million cases of poisoning, resulting in 220,000 deaths, occur annually worldwide, with the vast majority (99%) of these cases occurring in developing nations.

While previous estimates have suggested that the number of pesticide poisoning deaths is around 220,000, these numbers may be underestimated, as more recent studies suggest the actual number of deaths may be closer to 300,000. Shockingly, of these deaths, 175,000 occur annually in China alone [3]. Effective measures must be implemented to reduce the number of pesticide poisoning incidents in developing countries to prevent needless loss of life.

The deleterious effects of pesticide toxicity on public health cannot be overstated, as it is a major contributor to morbidity and mortality worldwide. Developing nations, especially those in the Asia-Pacific region, bear this burden, with an estimated 95% of lethal pesticide incidents occurring in these regions [4].

In Sri Lanka, acute pesticide poisoning poses a significant challenge to public health, particularly in certain agricultural regions. Pesticide poisoning has surpassed all other causes of death in government hospitals in these areas. Notably, intentional pesticide poisoning, often as a means of suicide, is the leading cause of this morbidity and mortality, affecting predominantly young adult males. While occupational exposure to pesticides also causes poisoning, it is less well-documented. Nevertheless, high rates of severe pesticide poisoning have been observed in irrigation zones of Sri Lanka, with 68% of cases resulting from the intentional ingestion of liquid pesticides. The ready availability and widespread use of highly toxic pesticides is believed to be the primary driver of this epidemic [5].

Nepal, a low-middle-income country (LMIC) in South Asia with a population of approximately 29 million, relies significantly on agriculture. However, this demographic is confronted with a self-poisoning with pesticides is responsible for 14% to 20% of global suicides, resulting in an estimated 110,000 to 168,000 deaths annually. Poisoning is a prevalent method of suicide in Nepal, and pesticides are the most frequently used poison [6-8].

This study delves into the scientific publications on pesticide poisoning in South Asian countries, specifically identifying the countries that have produced the highest research volume. The results of this study can provide valuable insights and help researchers, policymakers, and other stakeholders to understand the current state of research on pesticide poisoning in South Asia. The findings can also inform the development of research agendas, policies, and interventions to address the issue of pesticide poisoning in the region. Furthermore, this study can be useful for researchers and scholars researching pesticide poisoning in South Asia. The bibliometric analysis can help them identify key research themes, gaps, and opportunities for future research. Overall, this bibliometric analysis can advance knowledge on pesticide poisoning in South Asia and help to improve public health outcomes by providing evidence-based information for decision-making and policy development.

Despite their limitations, bibliometric studies have inherent value in the scientific community. They serve as a tool to facilitate discussion and offer a comprehensive overview of significant scientific research published in recent years, thereby revealing patterns, themes, and trends in the literature. This bibliometric analysis provides a useful perspective for individuals actively involved in the pesticide poisoning literature, practitioners, or trainees. While it may not encompass the earliest publications, it highlights the scientific research about pesticide poisoning in South Asian countries. The insights provided by such an analysis can prove invaluable in furthering our understanding of the topic and developing more effective strategies to address the issue.

## Review

Materials and methods

Study Setting and Design

The bibliometric search was carried out utilizing the PubMed advanced search engine. PubMed is widely recognized for providing a standard dataset, which facilitates bibliographic analysis and tracking of essential criteria such as author names, keywords, affiliations, countries, journal titles, number of citations, and broad subject areas. The PubMed core collection was searched from 2000 to 2022, enabling the acquisition of pertinent data for the current bibliometric analysis.

Search Strategy

In bibliometric analysis, a crucial aspect is to devise a dependable search query that can maximize the number of relevant publications while minimizing the occurrence of false-positive outcomes. This study aimed to collect comprehensive scientific publications on pesticide poisoning in South Asian countries by formulating a highly reliable search query. The authors utilized Medical Subject Heading (MeSH) terms from PubMed to create a search strategy that incorporated the following keywords: "Poison," "Toxicant," "Insecticide," "Herbicide," "Fungicide," "Toxic," "Germicide," "Biopesticide," "Acaricide," "Toxin," and "Microbicide." The search was specifically limited to the South Asian region and encompassed nine countries: Afghanistan, Bangladesh, Bhutan, India, Iran, Maldives, Nepal, Pakistan, and Sri Lanka. The accuracy of the search strategy was confirmed through a meticulous manual review of the obtained results.

Statistical Analysis

We investigated the records of the articles utilizing R Studio 2021 and Microsoft Excel 2019, which are designed explicitly for data analysis purposes and have attained recognition within the scientific community. Our analysis involved gathering data from the PubMed database, which we presented in a tabular format. The tabulation of data, including creating a trend graph illustrating the publication volume over time, was completed using Microsoft Excel 2019.

Data Extraction

A team of two authors developed the search methodology and extraction of literature and bibliometric indicators. The number of scientific publications, country-level articles, and the most relevant sources were extracted utilizing an appropriate analysis technique. The data was then analyzed using relational figures and tables. The bibliometric analysis comprised two steps. The first step involved the examination of the annual scientific output and collaboration patterns among nations, organizations, and authors. In the second step, we studied the geographical distribution and trends of journals, countries, institutions, and authors.

Results

Analysis of Annual Scientific Production

A comprehensive search was conducted on the PubMed database to collect 417 scientific research publications on pesticide poisoning in South Asian countries. The time frame for the search was set from 2000 to 2022, and the publications were obtained from 166 unique sources. As depicted in Figure 1, the annual scientific production on this topic peaked in 2017, with 40 publications. Furthermore, there was a noticeable escalation in the annual growth rate of research articles following 2014. These trends suggest an increasing focus on scientific investigation of pesticide poisoning in South Asian countries.

**Figure 1:** A graphical representation of the annual scientific production from 2000 to 2022.

The Productivity of the Leading Authors Over a Period

A compilation of the foremost 10 authors was generated. A comprehensive analysis of these leading authors and their output patterns over time illuminated that Acharya NR was the most prolific author between 2008 and 2021. This period witnessed Acharya NR produce a total of 17 articles, as demonstrated by Figure 2.

**Figure 2:** A graphical representation of the annual production analysis of the top authors over time.

Analysis of the Most Relevant Source

According to the findings illustrated in Figure 3, the preeminent scholarly journals, as determined by publication count, are *PLoS One* and *PLoS Neglected Tropical Diseases*. These journals have the highest number of published works. The *American Journal of Tropical Medicine and Hygiene* and the *Tropical Medicine and International Health* are closely behind, each with 16 publications.

**Figure 3:** A graphical illustration of the most relevant source with their article frequency.

Analysis of Country-Wise Scientific Production

Figure 4 represents the number of scientific publications generated by various Asian nations. As per the data, India has emerged as the leading country in scientific publications, producing a staggering 770. This is followed by Iran at 291 and the United States at 246. Other countries such as Bangladesh, Nepal, Pakistan, Thailand, Sri Lanka, the UK, and Australia have also contributed to the scientific literature with respective outputs of 157, 115, 99, 86, 76, 76, and 43 publications.

**Figure 4:** A graphical illustration of the country-wise scientific production.

Discussion

Bibliometric analysis is a widely utilized method for evaluating scientific publications, encompassing qualitative and quantitative approaches involving disseminating and utilizing published material. Typically, bibliometric studies reveal global research trends in a particular subject area, discipline, institution, or country [9].

Poisoning represents a significant clinical and public health problem in LMICs, particularly in India, despite often being neglected [1]. The issue of underreporting, including deficient death certification procedures and social stigma regarding suicide, persists. The limited availability of clinical and laboratory services for accurate diagnosis only compounds the issue. Despite these limitations, the Indian literature indicates a distressing incidence of deaths, predominantly attributed to intentional pesticide poisoning. Such data highlights the imperative for regulating highly hazardous pesticides (HHPs), as recommended by the World Health Organization (WHO) and the Food and Agriculture Organization (FAO), to prevent these fatalities [10-11].

As per the data provided by the Indian police, in 2015, more than 20,000 Indian citizens succumbed to self-inflicted poisoning from pesticides. Despite a consistent escalation in suicide rates since 1981, the overall rates of pesticide and general suicides have exhibited only marginal fluctuations in India since 2001. This pattern diverges significantly from neighboring countries such as Sri Lanka and Bangladesh, where the rates of both total and pesticide-induced suicides have significantly declined following the regulation of pesticides and the discontinuation of HHPs from national agricultural practices [12].

## Conclusions

Based on the findings of our study, it is evident that there has been a noteworthy increase in research efforts about pesticide toxicity in recent years. This is particularly evident in South Asian countries, where India has demonstrated higher scientific publication productivity than other nations. To further advance our understanding of pesticide poisoning and its associated health risks, it is essential to encourage and facilitate collaborative research projects among international teams. Such initiatives can help overcome barriers to information sharing and promote the synthesis of knowledge gleaned from diverse research contexts. By pooling resources, expertise, and data, researchers can better elucidate the mechanisms of pesticide toxicity, identify effective prevention and intervention strategies, and promote the development of safer, more sustainable pest management practices. In doing so, we can better protect human health and environmental well-being from the harmful effects of pesticides, both now and in the future.
